This article has been retracted.

# Correlation Analysis of Vaspin Gene Polymorphisms and Polycystic Ovary Syndrome Based on Intelligent Medicine

**DOI:** 10.1155/2022/6154233

**Published:** 2022-05-16

**Authors:** Yingjie Tang, Ting Huang, Yingzheng Pan

**Affiliations:** Department of Obstetrics and Gynecology, Chongqing Health Center for Women and Children, Chongqing 401147, Chongqing, China

## Abstract

Polycystic ovary syndrome (PCOS) is now a common gynecological endocrine disease, also known as Stein–Leventhal syndrome. Studies have found that Vaspin gene polymorphism is significantly associated with diabetes and cardiovascular disease, and PCOS has a clear glucose metabolism abnormality. So far, because the cause of PCOS is not clear, many problems such as the etiology, diagnostic criteria, prevention, and treatment of PCOS remain unsolved. Which also makes PCOS attract the attention of academic circles. Therefore, it is urgent to clarify the pathogenesis of PCOS, in order to explore the clinical correlation between the polymorphism of the Vaspin gene and polycystic ovary syndrome. This article introduces the correlation analysis study of Vaspin gene polymorphisms and polycystic ovary syndrome based on intelligent medicine. This article first selected 40 patients with PCOS as the experimental group and then selected 40 patients without PCOS as the control group. Secondly, through the detection methods of hs-CRP level detection and oil red O fat staining and passed two sets of control experiments. Finally, intelligent medical data analysis was used to analyze the location of the Vaspin gene in the experimental group and the control group. The final result showed that the correlation reached 75%.

## 1. Introduction

### 1.1. Research Background and Significance

A medical diagnosis and treatment expert system (ES) is a computer program system with a large amount of medical knowledge and disease diagnosis experience in specific medical fields. The system provides doctors with various medical knowledge, reasoning experience, and possible conventional diagnosis and treatment schemes at any time and plays an auxiliary role of “extending human brain memory” and “doctor assistant.” In particular, it can help doctors in grass-roots areas who are young and lack of clinical experience to improve the reliability of diagnosis results and optimize diagnosis and treatment plans. Polycystic ovary syndrome is a common and highly complex endocrine disorder and metabolic disorder. The incidence rate is gradually increasing, and the incidence rate is 6–10% in women of childbearing age [1, 2], while in the anovulatory type the incidence of infertility patients reaches 30–60% and is even reported as high as 70% [3]. The clinical phenotype of PCOS is heterogeneous, characterized by menstrual disorders, infertility, hirsutism, acne, obesity, and acanthosis nigricans. In addition to showing reproductive dysfunction, with age and endometrial cancer [4, 5]. Therefore, the impact of this disease is not limited to the childbearing age, it seriously affects the patient's physical and mental health and even affects family harmony. The exact pathogenesis of PCOS is still unclear. It is generally believed that PCOS is a disease caused by multiple factors such as heredity, environment, and lifestyle [6]. For PCOS, a complex and multicause disease, there are more than 100 PCOS susceptibility genes reported, including genes involved in the synthesis or mediation of steroid hormones, such as androgen-related genes, and metabolism-related genes, such as insulin growth factors and obesity genes. There are genes related to chronic inflammation [7]. But it did not work, as in the study of [8]. The genetic material and cyclic Vaspin factor Hida used differential screening technology in the visceral adipose tissue of the spontaneous type 2 diabetes obese rat model to isolate an adipokines similar to the serine inhibitor superfamily [9]. It has insulin sensitization and is also involved in the biological activities of glucose and lipid metabolism, inflammation, and other biological activities. Most studies have shown that Vaspin is closely related to insulin sensitivity and obesity [10, 11]. Based on the above-given theory, this provides a new research direction for PCOS. What is the specific relationship between Vaspin adipokines and PCOS patients? Is there an abnormal expression of Vaspin adipokines in PCOS patients? Is it related to other metabolic abnormalities in PCOS patients? The theoretical basis for the diagnosis and treatment of PCOS in the future needs to be further studied. In this experiment, by studying the expression of Vaspin adipokines in PCOS patients and control groups and the correlation between Vaspin adipokines and indicators of glucose and lipid metabolism and sex hormone metabolism in PCOS patients, the role of Vaspin adipokines in the pathogenesis of PC0S was explored, to provide a basis for future clinical work [12, 13]. In this paper, Vaspin gene polymorphism of intelligent medicine is applied to the correlation analysis of polycystic ovary syndrome, which has certain innovation and clinical value.

### 1.2. Related Content

Polycystic ovary syndrome is a common endocrine disease that affects approximately one-fifth of women worldwide. Liu designed the 160 individuals in the experimental study to be divided into 2 groups. His research uses ELISA to detect serum IL6 and uses TaqMan allele discrimination analysis technology to analyze the HSD11B1rs12086634(T/G) polymorphism [1]. Serum IL6 in PCO patients increased, and the frequency of GG and TG genotypes increased [14]. Dogan et al. assesses the association between insulin resistance in PCOS patients [15]. He set 87 PCOS women, 48 obese, and 39 normal weights as the experimental group. After the measurement, he compared the experimental group with the nonPCOS group, and the plasma Vaspin level of PCOS patients was significantly reduced [16]. Moreover, Vaspin thinks in the nonPCOS group, there was a negative correlation between plasma Vaspin level and body weight, so he predicted that the occurrence of PCOS was related to the decrease in the Vaspin level. The effect of nutritional status on Vaspin levels that he observed in nonPCOS women was subsequently eliminated, possibly due to more severe insulin resistance. Sharma P discussed the relationship between the VDR gene and the polymorphisms of AMH and AMHR2 genes (Apa1, Bsm1, Fok1, and Cdx2) and their influence on the levels of AMH and 25(OH)D in women with PCOS [17]. In the end, his experimental results of VDR Cdx2 polymorphism analysis showed that compared with the control group, the frequency of homozygous GG mutant genotypes in the PCOS group was significantly higher in the experimental group [18]. However, the shortcomings of these studies lie in the insufficient consideration of some performance and reference data.

### 1.3. Main Content

The main content of this article is to select patients with PCOS as the experimental group and select normal people without the disease as the control group. The experimental data are tested by the experimental method of hs-CRP level detection and oil red O fat staining, and finally obtained experimental data after data analysis through the intelligent Internet of Things, it is concluded that the Vaspin gene polymorphism site has a strong clinical correlation with polycystic ovary syndrome.

## 2. The Application of Smart Medical Care and the Calculation Method of Medical Data

### 2.1. Intelligent Medical

Intelligent medical care is to gradually reach informationization by creating a regional medical information platform for health records and using the most advanced Internet of Things technology to achieve interaction between patients and medical personnel, medical institutions, and medical equipment. In the context of the new medical reform, intelligent medical care is coming into the lives of ordinary people. With increasing life expectancy, declining birth rates, and health concerns, people in modern society need better healthcare systems. Thus, telemedicine and e-health are urgently needed. With the help of IoT/cloud computing technology, artificial intelligence expert system, and intelligent devices of embedded systems, a perfect IoT medical system can be built, so that all people can enjoy the top medical service equally and solve or reduce the phenomenon that the lack of medical resources leads to the difficulty of seeing the doctor, the tension between doctors and patients, and the frequent occurrence of accidents. The regional health information system diagram is shown in Figure 1.

As shown in Figure 1, the regional health information system includes inspections, inspection prompts, treatment safety warnings, expert remote consultation and consultation, expert outpatient appointments, and electronic disease detection. These functions can form smart medical care for community medical care, two-way referral, and health management. Therefore, this paper builds a data analysis model through intelligent medical care.

### 2.2. Calculation of Medical Knowledge Base

When estimating the distribution of a random variable, the main basis is the distribution in its sample. In order to solve this problem, it is necessary to add a prior distribution. Without any redundant knowledge, the simplest prior distribution is the average distribution. The value of *Z* is 10.

(1) $$\begin{array}{c} Y\left(d_{n}\right)=\frac{\left(fd_{n}\right)}{\sum \left(fd_{n}+Z\right)}. \end{array}$$

In the diseases and symptoms, similar to disease, the formula for calculating symptoms is as follows:

(2) $$\begin{array}{c} P\left(s_{n}\right)=\frac{\left(fs_{n}+Z\right)}{\sum \left(fs_{n}+Z\right)}. \end{array}$$

Here, *Fsd* is the number of times that disease *j* and symptom *n* appear together, and the value of *Z* is 10.

(3) $$\begin{array}{c} P\left(s_{n}|d_{j}\right)=\frac{\left(fs_{n}d_{j}+Z\right)}{\sum fs_{n}d_{j}+Z}. \end{array}$$

In the disease and gender, first of all, gender has its own prior ratio. *Fg* represents the number of occurrences of gender.

(4) $$\begin{array}{c} P\left(g_{n}\right)=\frac{fg_{n}}{\sum fg_{n}}. \end{array}$$

In the case that a certain disease has been changed, the probability of gender is the following formula:

(5) $$\begin{array}{c} P\left(g_{n}|d_{j}\right)=\left(fg_{n}d_{j}+\frac{Z}{\sum fg_{nd_{j}+Z}}\right). \end{array}$$

Similarly, age has a prior probability, and the calculation formula is as follows:

(6) $$\begin{array}{c} P\left(g_{n}\right)=\frac{fg_{n}}{\sum fg_{n}}. \end{array}$$

In the case of already suffering from a certain disease, the probability formula of age is as follows:

(7) $$\begin{array}{c} P\left(g_{n}|a_{j}\right)=\left(fg_{n}a_{j}+\frac{Z}{\sum \left(fg_{n}a_{j}+Z\right)}\right). \end{array}$$

The goal of this part is to mine the list of entities in the knowledge base and the appearance frequency of entities from a large amount of data, as well as the relationship between entities and attributes, and the strength of the relationship between different entities. In order to achieve the purpose of knowledge base mining, a very important task is how to identify entities from the data. Here, according to the different types of data, different methods need to be adopted.

### 2.3. Difficulties in Smart Medical Analysis

#### 2.3.1. Intelligent Medical Analysis

This article summarizes the manifestations of implicit errors in smart medical care into the following two forms:

*(1) Functional Redundancy*. The behavior trajectory of smart medical care will not be deadlocked, but redundant functions will appear. For example, in the intelligent nursing system, when the monitor senses that the patient's vital characteristics are different, an alarm is issued; however, due to the participation of the role of the nurse in the medical environment, the system has a certain degree of randomness, and multiple nurses receive the alarm. The treatment will not cause errors in the operation of the intelligent nursing system and the system will not deadlock, but for the patient, the medical experience is uncomfortable, and in addition, related medical resources are wasted.

*(2) Loss of Function*. Due to the lack of some functions in the analysis process of intelligent medical treatment, the efficiency of data analysis is low. For example, in the intelligent nursing system, the function assignment of nurses does not have a transfer function and a certain nurse has a heavy workload, but other nurses are idle, resulting in low efficiency. Some of these errors can be coordinated through appropriate management methods when the system process is actually running, but it may be more efficient if possible problems are discovered and avoided during the design phase. Moreover, the medical environment is diverse, random, and changeable. In different medical environments, the process of the medical system is different, and the medical system is applied to the specific professional field of medicine. The professional knowledge of the system designer may not be sufficient. Therefore, it is difficult for the system designer to predict all errors based on experience and consider the system design thoroughly.

#### 2.3.2. Benefits of Intelligent Medicine

An intelligent medical aided diagnosis system is an intelligent computer program. Its intelligence is reflected in its ability to use medical knowledge to simulate the reasoning process of medical experts in diagnosing diseases and give reasonable disease treatment plans, which can help doctors with poor basic medical levels to solve complex medical problems. The perfect medical knowledge base integrates the medical knowledge of various disciplines in the medical field. The expert diagnosis system using the knowledge base can even surpass a single medical expert; and, the system will not affect the judgment of the disease due to subjective factors such as fatigue or pressure like human experts, so as to reduce the misdiagnosis rate and missed diagnosis rate.

Expert system structures in different fields should be designed in combination with specific application fields and tasks to be handled. However, no matter which design structure must meet the two requirements of storing domain knowledge and solving problems with knowledge. Therefore, the knowledge base used to store domain knowledge and the inference engine using knowledge for reasoning are indispensable functional modules of the system.

## 3. Intelligent Medical Method Analysis and Experimental Procedures

### 3.1. Analysis of the Main Components Based on the Intelligent Medical Internet of Things

#### 3.1.1. Principal Component Analysis

Principal component analysis, also called principal component analysis, is a statistical technique based on dimensionality reduction methods. The principle is to transform a large number of original variables into a new set of variables that are not related to each other after processing, and the recombined variables can reflect the information of the original variables. Analytical knowledge varies according to the way it is obtained, and now text analysis methods based on statistical machine learning are usually used to analyze text. The main purpose of the principal component analysis is to use a small number of variables to explain the original large number of variables. The analysis steps of principal components are as follows:

(1) Data standardization:

(8) $$\begin{array}{c} Y_{ij}=\frac{x_{ij}-x_{j}}{Z_{j}}. \end{array}$$

Among them,

(9) $$\begin{array}{c} x_{i}=\frac{\sum_{i=1}^{n}x_{ij}}{n},\\ Z_{j}=\frac{\sum_{i=1}^{n}\left(x_{ij}-x_{j}\right)}{n-1}. \end{array}$$

(2) Calculate the correlation coefficient matrix:

(10) $$\begin{array}{c} P=\left[r_{ij}\right]xp. \end{array}$$

(3) Solve the matrix to determine the number of principal components:

(11) $$\begin{array}{c} \left|P-\gamma I=0\right|, \end{array}$$

(12) $$\begin{array}{c} \frac{\sum_{j=1}^{m}j}{\sum_{j=1}^{p}i}\geq 0.77. \end{array}$$

Solve (11) to obtain the characteristic roots of the equation and determine the value of *m* in (12).

(4) Principal component generation:

(13) $$\begin{array}{c} U_{ij}=Z_{i}bj. \end{array}$$

Among them, *U*1, *U*2, and *U*3 are the first, second, and third principal components, and so on, *Um* is the *m*-th principal component.

#### 3.1.2. Multilayer Perceptron

The multilayer perceptron is a multilayer feedforward neural network model. It is a network formed by adding a hidden layer to a neural network composed of a single layer of neurons. There are several definitions of hidden layers. The definitions used in this paper are as shown in the figure. Except that the output layer is not included in the hidden layer, other network hierarchies containing neurons are regarded as hidden layers. When an input signal enters, the first hidden layer first obtains the data of the input signal. After the signal is processed by the neurons of the first hidden layer, the generated output is transmitted to the next hidden layer and then to the output of the whole neural network at one time. It uses a back-propagation (BP) algorithm. The multilayer perceptron was originally used for classification, and then it can also be used for logistic regression. It can map data to a linearly separable hidden layer to achieve nonlinear data classification. The structure of the multilayer perceptron is shown in Figure 2.

Figure 2 shows the structure of a multilayer perceptron (MLP), which has two hidden layers. The network is fully connected, that is, except for the input layer (the input layer actually has no neurons, but input data) and the output layer, the neurons between any two adjacent layers are connected to each other.

### 3.2. Experimental Materials and Procedures

#### 3.2.1. Research Object

Experimental group: 40 PCOS patients were randomly selected, including 16 cases of O blood type, 9 cases of A blood type, 1 case of B blood type, and 1 case of AB blood type, with an average age of 24.60 ± 4.68 years. There was no blood relationship among the subjects in the group, and the experimenters all gave informed consent. Control group: 40 normal women were randomly selected as a healthy control group, including 14 cases of O blood type, 5 cases of A blood type, 10 cases of B blood type, and 11 cases of AB blood type, with an average age of 23.35 ± 3.52 years. Healthy control women should meet: ① regular menstruation and a menstrual cycle of 23–35 days; ② six sex hormone tests are normal; ③ transvaginal ultrasound examination of the uterus and bilateral ovaries shows no organic lesions and no polycystic ovaries.

*(1) Case Group Inclusion Criteria*. Age 18–40 years old, the diagnostic criteria refer to the Rotterdam diagnostic criteria.

*(2) The Inclusion Criteria of the Control Group*. Age 18–40, menstrual cycle 21–35 days, normal ovulation function, no history of adverse pregnancy, at least one or more normal birth history.

*(3) Sub-group*. The degree of IR is evaluated by the homeostatic model insulin resistance index (HOMA-IR), HOMA-IR = fasting blood glucose *∗* fasting insulin 22.5; HOMA-IR ≥1.66 is judged as IR. The cases were divided into 29 cases in the PCOS-IR (insulin resistance) group and 16 cases in the PCOS-NIR (noninsulin resistance) group.

According to the WTO obesity standard BMI >25, they were divided into the overweight group and the nonobese group. Patients with BMI >25 de PCOS were divided into overweight and obese groups according to 25 < BIM < 30.

According to the different genotypes of the Vaspin gene A66G locus, C677T locus, and A1298C locus, three subgroups were classified: CC genome, CT genome, and TT genome; AA genome, AC genome, and CC genome; and AA genome, AG genome, and GG Genome.

*(4) PCOS Diagnostic Criteria*. The criteria in this article are based on the PCOS diagnostic criteria modified by the Rotterdam Conference in the Netherlands (the eighth edition textbook of gynecology). The PCOS diagnostic criteria are shown in Table 1. If at least 2 of the following 3 items are met, it is diagnosed as PCOS.

*(5) Collection of Blood Specimens*. All patients in the PCOS group and the control group have fasted for 7–11 hours, and after a 40-minute rest the next morning, blood was drawn from the vein. At the same time, keep 10 ml of venous blood, EDTA anticoagulant and store in the refrigerator at −40°C for genetic polymorphism detection.

*(6) Sampling*. All subjects in this study took 5–7 ml of cubital venous blood on an empty stomach and placed it in a 5 ml human venous blood anticoagulation tube containing ethylenediaminetetraacetic acid-2 sodium and numbered the anticoagulation tube according to the number of the research subject questionnaire. Make sure the numbers are consistent and stored at −80°C. The questionnaire includes name, age, ethnicity, marriage history, height, weight, waist circumference, hip circumference, systolic blood pressure, diastolic blood pressure, occupation, blood type, eating habits, course of disease, and family history. This article is based on symptoms and signs (age at menarche, menstrual disorders during menstruation, weight change trends, etc.), ovarian ultrasound examination, fasting blood glucose, insulin, sex hormones, total cholesterol, triglycerides, and other biochemical indicators.

#### 3.2.2. Research Methods

*(1) Anthropometric Examination*. Collect anthropometric parameters of all study subjects, including age, height, weight, waist circumference (WC), and hip circumference (HC), calculate body mass index (BMI) = weight (kg)/height 2 (m^2^), WHR = waist circumference hip circumference (cm). Waist measurement: the horizontal length from the navel to the waist. Hip measurement: the horizontal length of the most protruding part from the hip to the back.

*(2) Oil Red O Fat Stain*. The cells were seeded in a 6-well culture plate with sterile coverslips for culture, and PMA was used to induce the cells to transform into macrophages for 15–20 minutes, then the cells were washed with PBS solution, and the washing was repeated 4 times. Carry out oil red O fuel coloring in sequence, place in a 60°C oven for 15 minutes in the dark, and perform color separation with 60% isopropanol for a few seconds, then wash with deionized water 4 times, 2∼4 min each time and counterstain with hematoxylin for 2∼3 min, wash with deionized water again for 15 min, 1% hydrochloric acid alcohol color separation for 2∼3 s, then the water turns blue, microscope observation, the lipid in the image shows red particulate matter.

*(3) hs-CRP Level Detection*. The sensitized latex enhanced immunoturbidimetric method is used for detection, and the immunoturbidimetric method is used to detect the content of high-sensitivity C-reactive protein. The sample is combined with the particle-bound C-reactive protein antibody to form an antigen-antibody complex, resulting in suspended particles in the solution. Enhancement, the enhancement ratio is proportional to the concentration of high-sensitivity C-reactive protein in the sample. The detection steps are shown in Table 2.

As shown in Table 2, prepare 3 ul distilled water empty tube, distilled water calibration tube and sample tube are not prepared, prepare 3 ul calibration solution, sample tube is also 3 ul, then reagent 1 prepare empty tube table 300 ul, calibration tube 300 ul, sample tube 300 ul, mix and shake well, and then add reagent 2. The preparation of reagent 2 is also the empty meter tube 80 ul, the calibration meter 800 ul, and the sample tube 80 ul. Then, mix and shake well.

#### 3.2.3. Detection of Genetic Polymorphism

*(1) Main Instruments and Manufacturers*. The instruments and manufacturers used in this study are shown in Table 3.

*(2) PCR Amplification*. The amplification system is shown in Table 4.

PCR amplification conditions are 95 degrees celsius predenaturation for 10 minutes and 95 degrees celsius denaturation for 20 s. Then, 60 degrees celsius extension for 60 s. A total of 20 cycles, then 90 degrees celsius denaturation 30 s ⟶ 60 C extension for 90 s, a total of 30 cycles, PCR product at 4 Save in degrees celsius.

## 4. Experimental Results

### 4.1. Comparison of Anthropological Measurement Parameters between the Case Group and the Control Group

The comparison of anthropometric parameters between the case group and the control group is shown in Table 5. In this paper, 40 patients with polycystic ovary syndrome were selected from a municipal hospital as the experimental group, and then 40 patients with nonpolycystic ovary syndrome were selected as the control group. The average ages of the case group and the control group are about 25 years old and about 32 years old.

As shown in Table 5, in the parameter comparison between the PCOS group and the control group, the age of the PCOS group is 25 and the age of the control group is 32. The difference in age is still large, but it has no effect on the progress of the experiment. It is mainly to compare illness and disease-free, and the difference in age is not significant; in the PCOS group, the height is 1.58, and the height of the control group is 1.59, and there is no significant difference in height; in the weight, the weight of the PCOS group is 52 kg, and the control group's weight was 51 kg, and there was no significant difference in body weight; in BMI, the BMI of the PCOS group was 20.95, the BMI of the control group was 20.82, and there was no significant difference in BIM. Finally, in the comparison of waist circumference and hip circumference, the waist-to-hip ratio was mainly seen through comparative analysis. The WHR of the PCOS group was 0.86, and the WHR of the control group was 0.80. The difference in WHR was small, but the WHR of the PCOS group was higher. In summary, there is no significant difference in height, weight, and BMI, but there are some differences in WHR.

### 4.2. Vaspin Promotes Lipid Metabolism of Adipocytes

We first observed the effect of Vaspin on the formation of adipocyte-derived foam cells. Adipocytes were treated with Vaspin for 24 hours, and the lipid accumulation in the cells was observed by oil red O staining. The results showed that the red lipid droplets in the cells of the Vaspin treatment group were more obvious than those of the control group. The reduction, as shown in Figure 3, shows that Vaspin can significantly promote the outflow of cholesterol in fat cells, reduce lipid accumulation, strengthen lipid metabolism, and inhibit the formation of foam cells.

As shown in Table 6, in BIM <25, Vaspin, FBG, and HOMA-IR in the PCOS group were significantly higher than those in the control group. In BIM >25, Vaspin, FBG, and HOMA-IR in the PCOS group were also significantly higher than those in the control group. And, there are statistical differences (*P* < 0.05).

It can be seen that Vaspin is positively correlated with BMI. Multiple stepwise regression analysis shows that WHR is an independent factor for low serum Vaspin levels, suggesting that Vaspin is closely related to abdominal obesity. Based on the above research results, it is speculated that Vaspin is closely related to obesity, especially in patients with abdominal obesity. It may be that the increase in body fat content stimulates the secretion of Vaspin in adipose tissue and compensatory participation in the occurrence of obesity. It may also be that the body in an obese state compensatory causes the increase in serum Vaspin expression in order to adapt to the needs of metabolic narcotics. Correlation analysis shows that Vaspin is only positively correlated with FBG. Therefore, it is speculated that serum Vaspin may play a role in the lipid metabolism of PCOS.

### 4.3. Comparative Analysis of Vaspin and hs-Crp Levels between Groups

Compared with the control group, the Vaspin and hs-CRP levels of the experimental groups of patients with different body mass indexes were significantly increased, and the differences between the groups were statistically significant (*P* < 0.05), and the Vaspin and hs-CRP levels of the experimental group of patients -CRP levels showed a rising trend, and the differences between the groups were statistically significant (*P* < 0.05). The specific results are shown in Figure 4.

Through Pearson correlation analysis, the analysis shows that the correlation coefficient of Vaspin and hs-CRP is 0.751, the absolute value is between 0 and 1, and it is a positive correlation, *P* value < 0.01, as shown in Figure 5.

Explore the relationship between Vaspin and hs-CRP development, so as to provide a theoretical basis for the diagnosis, prevention, and prognosis of polycystic ovary syndrome.

### 4.4. Analysis of the Difference between the Different Genotypes of the a1298c Site of the Gene a1298c and the Levels of Plasma Fat, Vitamin 12, And Hcy in the PCOS Group and the Control Group

As shown in Table 7 and Figure 6, the Vaspin gene A1298C locus and polymorphism did not affect plasma lipid and HCY levels. Studies have shown that plasma HCY levels are closely related to adverse pregnancy outcomes. In this study, in order to avoid the influence of potential abnormal maternity factors on the HCY level of the control group, healthy people with at least one or more normal childbirth history were selected, so they are older and PCOS patients are relatively young. Therefore, in the results of this study, there is a difference between ages. The case group is younger than the control group. There is also a difference in HCY levels between the two groups. The physiological HCY level increases with age, which just shows that there is HCY metabolism disorder in PCOS patients.

### 4.5. Vaspin Gene c677t Locus Genotype (Cc) Increases the Risk of PCOS, and Allele C Is a Genetic Susceptibility Gene for PCOS

The frequencies of the three genotypes CC, CT, and TT at the C677T locus of the Vaspin gene accounted for 58.2%, 36.4%, and 5.55%, respectively in the PCOS group. The frequencies of the C and T alleles were 76.4% and 23.6%, respectively; the allele C was in the PCOS group. The distribution frequency of the PCOS group (76.4%) was significantly higher than that of the control group (60.9%), and the difference was statistically significant (*X*2 = 5.626, *P* < 0.05). Allele C increased the risk of PCOS by 2.077 times. The type distribution and allele frequency distribution of the C677T locus of the Vaspin gene are shown in Figure 7.

## 5. Discussion

Polycystic ovary syndrome (PCOS) is an endocrine disorder syndrome with reproductive dysfunction and abnormal glucose metabolism. It is characterized by persistent anovulation, multiple follicle immaturity, hyperandrogenemia, insulin resistance, and polycystic ovary. It has clinical manifestations such as abnormal menstruation, hairiness, obesity, infertility, bilateral ovarian enlargement, and cystic changes.

PCOS is a common cause of the menstrual disorder and marital infertility in reproductive women. Due to different degrees of insulin resistance, the risk of atherosclerosis and cardiovascular disease in patients with PCOS is significantly increased. The incidence rate of PCOS is relatively high, which accounts for 5% to 10% of women of childbearing age. At present, the pathogenesis of the disease is not clear, which may be related to genetic, environmental, and other factors.

Vaspin is a serine protease inhibitor, first reported by Hida et al. In 2005. It belongs to the serine protease inhibitor family. It is found in visceral adipose tissue of spontaneous type 2 diabetes rat, also known as visceral adipose tissue derived serine protease, inhibiting ∼lJ (visceral adipose tissue derived serine protease inhibitor, Vaspin). Studies have found that Vaspin gene polymorphism is significantly associated with diabetes and cardiovascular disease L 3I. PCOS has clear abnormal glucose metabolism. Therefore, this study aims to judge the relationship between Vaspin gene polymorphism and PCOS.

## 6. Conclusions

In this paper, through the comparative analysis of the experimental group and the control group, and then through the human body detection method, hs-CRP level detection, and oil red O fat staining for detection, the finally obtained experimental data are analyzed through the intelligent Internet of Things, and the following results are obtained in conclusion. First, Vaspin may play a role in the lipid metabolism of PCOS. Second, explore the correlation between the development of Vaspin and hs-CRP, so as to provide a theoretical basis for the diagnosis, prevention, and prognosis of polycystic ovary syndrome. Third, there is HCY metabolism disorder in PCOS patients. Fourth, the allele C of Vaspin increases the risk of PCOS. [19].

## Figures and Tables

**Figure 1:** Regional health information system.

**Figure 2:** Diagram of multilayer perception mechanism.

**Figure 3:** Oil red O staining to observe the effect of Vaspin on the lipid content of adipocytes.

**Figure 4:** Comparison of Vaspin and hs-CRP levels between groups.

**Figure 5:** Correlation between Vaspin and hs-CRP.

**Figure 6:** Comparison of HCY and lipids of different genotypes at the A1298C site in the control group.

**Figure 7:** The proportion of each parameter in the PCOS group and the control group.

**Table 1:** PCOS diagnostic criteria.

Disease	Pathological scope
Ovulation status	Sparse ovulation or anovulation

Clinical manifestations	The clinical manifestations of hyperandrogenemia and/or the biochemical manifestations of hyperandrogenemia

Ovarian polycystic changes	There are more than 12 follicles with a diameter of 2–9 mm in one or both ovaries, and/or the ovaries are 10 ml larger in volume

**Table 2:** hs-CRP detection steps.

Addition	Empty meter tube	Calibration tube	Sample tube
Distilled water	3	—	—
Calibration solution	—	3	—
Sample	—	—	3
Reagent 1	300	300	300
Mix well, then add reagent 2			
Reagent 2	80	80	80
Mix well and read the absorbance at 600 nm for 3 minutes to obtain the rate of change in absorbance per minute.			

**Table 3:** Major instruments and manufacturers.

Nucleic acid concentration analyzer	Manufacturer: United States
Clean bench	Manufacturer: Jinan
High-speed centrifuge	Manufacturer: Thermo Pioc
Pipette	Manufacturer: Eppendorf
Constant temperature water bath-dry thermostat	Manufacturer: Hangzhou
Vortex oscillator	Manufacturer: United States
PCR fluorescence quantitative analyzer	Manufacturer: Shanghai

**Table 4:** Amplification system.

DNA template	0.4 ul
Upstream/downstream primer	0.4 ul
Pfu enzyme	5 ul
ddH2O	4 ul
Total capacity	12 ul

**Table 5:** Comparison of anthropometric parameters between the PCOS group and the control group.

Variable	PCOS group	Control group (*r* = 46)	*t*	*P* value
Age	25	32.	−7.236	<0 001
Height (m)	1.58	1.59	−0.486	0.628
Weight (kg)	52	51	−0.16	0.987
BMI (kg M2)	20.95	20.82	0.212	0833
Waist circumference (am)	77.03	72.26	3.408	0.01
Hip circumference (am)	89	90	−0.835	0.406.
Waist/Hip (WHR)	0.86	0.80	6.192	<0.001

**Table 6:** Comparison of clinical parameters between normal weight and overweight in the PCOS group and the control group.

	BMI <25			BMI >25		
	PCOS group	Control group	*P*	PCOS group	Control group	*P*
Vaspin	0.657	0.452	0.036	0.875	0.564	0.041
FBG	8.915	0.248	0.000	9.204	5.889	0.000
HOMA-IR	3.584	3.459	0.037	13.048	3.654	0.006

**Table 7:** Difference analysis of plasma fat, vitamin 12, and HCY levels.

Group	Plasma fat			*F* value	*P* value
-	AA	AG	GG	-	-
PCOS group	18.45	23.55	15.01	1.097	0.345
Control group	21.78	25.68	35.64	0.872	0.488

Group	Plasma vitamins			-	-
-	AA	AG	GG	*F* value	*P* value

PCOS group	408.33	500.56	401.34	0.077	0.984
Control group	404.6	395.2	501.6	0.759	0.475

Group	HCY			-	-
-	AA	AG	GG	*F* value	*P* value

PCOS group	10.05	9.17	11.47	3.047	0.056
Control group	8.84	8.63	8.43	0.820	0.921

## Data Availability

The data used to support the study are included in the paper.
